The article "Ultrasound Evaluation of Pelvic Floor Function after Transumbilical Laparoscopic Single-Site Total Hysterectomy Using Deep Learning Algorithm" was published in 2022. Journal: Comput Math Methods Med.

# Ultrasound Evaluation of Pelvic Floor Function after Transumbilical Laparoscopic Single-Site Total Hysterectomy Using Deep Learning Algorithm

**DOI:** 10.1155/2022/1116332

**Published:** 2022-08-10

**Authors:** Yan Zhu, Jiamiao Zhang, Zhonglei Ji, Wen Liu, Mingyue Li, Enhui Xia, Jing Zhang, Jianqing Wang

**Affiliations:** ^1^Department of Obstetrics and Gynecology, The Yancheng Clinical College of Xuzhou Medical University, The First People's Hospital of Yancheng, Yancheng, 224001 Jiangsu, China; ^2^Department of Ultrasound, The Yancheng Clinical College of Xuzhou Medical University, The First People's Hospital of Yancheng, Yancheng, 224001 Jiangsu, China

## Abstract

This study was aimed at investigating the ultrasound based on deep learning algorithm to evaluate the rehabilitation effect of transumbilical laparoscopic single-site total hysterectomy on pelvic floor function in patients. The bilinear convolutional neural network (BCNN) structure was constructed in the ultrasound imaging system. The spatial transformer network (STN) was used to preserve image information. Two algorithms, BCNN-R and BCNN-S, were proposed to remove sensitive information after ultrasonic image processing, and then, subtle features of the image were identified and classified. 80 patients undergoing transumbilical laparoscopic single-site total hysterectomy in hospital were randomly divided into a control group and a treatment group, with 40 cases in each group. In the control group, conventional ultrasound was used to assess the image of pelvic floor function in patients undergoing laparoendoscopic single-site surgery (LESS); in the observation group, ultrasound based on deep learning algorithm was used. The postoperative incision pain score, average postoperative anus exhaust time, average hospital stay, and postoperative satisfaction of the two groups were evaluated, respectively. The highest accuracy of constructed network BCNN-S was 88.98%; the highest recall rate of BCNN-R was 88.51%; the highest accuracy rate of BCNN-R was 97.34%. The operation time, intraoperative blood loss, and exhaust time were similar between the two groups, and the difference had no statistical significance (*P* > 0.05). The numerical rating scale (NRS) scores were compared, the observation group had less pain, the difference between the two groups had statistical significance (*P* < 0.05), and the postoperative recovery was good. The BCNN based on deep learning can realize the imaging of the uterus by ultrasound and realize the evaluation of pelvic floor function, and the probability of pelvic floor dysfunction is small, which is worthy of clinical promotion.

## 1. Introduction

Pelvic floor disease is a degenerative lesion including urinary incontinence and pelvic organ prolapse [1]. In the United States, nearly 400,000 patients undergo surgery due to pelvic floor dysfunction each year, and 300,000 cases occur during hospitalization. Each year, 33% of women have different pelvic floor dysfunction (PFD) before the age of 60 and require hysterectomy [2]. Hysterectomy is closely related to PFD, which can improve the risk of postoperative pelvic floor dysfunction and affect the quality of life of patients [3]. The pelvic floor function of normal women mainly relies on intact muscle strength, nerves, and ligaments. The interaction of various organs allows the pelvic floor structure to reach a normal dynamic balance state [4]. The hysterectomy can damage the neural tissue, impair vascular nutrition, and severely destroy important supporting structures such as muscles, ligaments, fascia, and connective tissue [5, 6]. PDF in women is usually judged based on the patient's clinical symptoms as well as the corresponding examination results, and the examinations include finger pressure test, urodynamic examination, and magnetic resonance imaging, but these modalities have the disadvantage of poor reproducibility and cannot comprehensively evaluate the pelvic floor function of the anatomy for dynamic imaging, safety, and repeated procedures [7, 8]. At present, transperineal pelvic floor ultrasound is increasingly loved by researchers to evaluate the dynamic changes of pelvic floor function. Pelvic floor ultrasound enables real-time observation of pelvic anatomy and function and enables dynamic imaging, which has become a major modality for assessing pelvic floor ultrasound [9, 10].

Transumbilical laparoendoscopic single-site surgery (TU-LESS) is a surgical technique performed using surgical instruments through the pore channel, mainly using the umbilicus to place multiple operating pore channels as well as the operating platform of the laparoscope in the abdomen, which can reduce abdominal infections caused by gastrointestinal tract as well as transapproach surgery, with the characteristics of mild pain, rapid recovery, no earthworm-like scar left in the abdomen, safety, and minimal invasion. In this process, it can also use the natural wrinkle site of the umbilicus to cover the surgical incision, which can meet the requirements of women for abdominal “scarless” cosmetology [11, 12]. Compared with traditional multiport laparoscopy, TU-LESS is easier to perform in total hysterectomy, can shorten gastrointestinal recovery time and postoperative ambulation time, and can remove the uterus through a single port at the umbilicus and through an approach in a manner similar to “apple cutting.” “Chopstick effect” between instruments is one reason for prolonged operation time [13, 14].

With the advantages of high sensitivity, noninvasion, easy operation, and low cost of ultrasound imaging, real-time three-dimensional (four-dimensional) ultrasound imaging has become an effective diagnostic tool in imaging systems in the 21st century [15]. Ultrasound is widely used in obstetrics and gynecology without ionizing radiation, cost-effective, and easy to approach, for example, abdominal ultrasound, cardiovascular ultrasound, electrocardiogram, and prenatal diagnostic ultrasound, but the presence of pseudonoise in ultrasound imaging causes reduced imaging quality and is also a challenge in ultrasound; relying only on the experience of doctors, as well as the proficiency of operators, there are significant differences in results in different institutions as well as different ultrasound systems [16, 17]. This requires the use of advanced intelligent ultrasound image analysis algorithms to intervene imaging quality. Deep learning technology has made it successful for natural image recognition in the construction of large-scale image datasets, and high-resolution ultrasound imaging equipment has accumulated many ultrasound image data, which also makes deep learning possible for the auxiliary diagnosis of images [18, 19]. The bilinear convolutional neural network (BCNN) enables a good classification of images [20]. Yosinski et al. [21] pointed put when learning the features of the underlying CNN that the CNN network can get distinct features with increasing depth, and the closer to the input end, the more specific information the feature displays.

The ultrasonic transverse section of patients with total hysterectomy was identified, and the BCNN was used to identify the ultrasonic transverse section of the uterus.

The innovation is that the intelligent algorithm is used to identify high resolutely the transverse section, and the extracted features are fused, which is helpful to retain the subtle features. It is hoped that it can provide reference for ultrasound evaluation of pelvic floor function in patients with transumbilical laparoscopic single-site total hysterectomy and provide theoretical basis for clinical work.

## 2. Materials and Methods

### 2.1. Subjects

Eighty patients admitted to hospital from June 2018 to June 2020 who underwent transumbilical laparoscopic single-site total hysterectomy were selected. The age of the study subjects ranged from 32 to 50 years, with an average of 42.5 ± 3.61 years and BMI of 23.67 ± 1.2 kg/m^2^. There were 28 cases of uterine fibroids, 19 cases of endometrial lesions, and 33 cases of adenomyosis. The patients were randomly divided into the control group (*n* = 40) and the treatment group (*n* = 40) by random number table method. There was no significant difference in basic information between the two groups (*P* > 0.05). Preoperative gynecological examination of the uteri was less than 4 months of gestation with good range of motion, and the operation was completed by the same physician. This study had been approved by the ethics committee of the hospital, and the patients and their families signed the informed consent form.

Inclusion criteria: patients with uterine fibroids or adenomyosis diagnosed by routine cervical biopsy or cervical liquid-based cytology before surgery; patients with complete clinical data; patients without cervical malignant lesions or uterine prolapse; patients without fertility requirements, nonpregnant patients; patients without serious medical and surgical diseases and a history of repeated surgery.

Exclusion criteria: patients who are allergic to the drugs used; patients who are critically ill and unable to cooperate; patients with chronic diseases such as heart, brain, liver, and kidney; patients with mental diseases; patients with systemic infection.

### 2.2. Treatment Methods

Ultrasonic diagnostic apparatus was used. The intestinal tract of the patient with the probe frequency of 4-8H was emptied, the patient laid on the examination bed, and the probe coated with coupling agent and covered with disposable film gloves was placed at the perineum to clearly show the uterine condition. In the Valsalva state and at rest, distance from the bladder neck to the posteroinferior border of the pubic symphysis (BNSD), distance from the external cervical orifice to the posteroinferior border of the pubic symphysis (CSD), posterior urethrovesical angle (PUA), and bladder neck mobility and the difference in the distance from the bladder neck to the posteroinferior border of the pubic symphysis (BND) under the maximum Valsalva state and at rest were compared between two groups. For measurements in both states, all data were measured in triplicate by 3 examining physicians and then averaged.

The patient was anesthetized by endotracheal intubation. The bladder lithotomy position was taken, and the uterine lifting device was placed. The patient's posture was low head and high foot. The longitudinal incision (about 10 mm) was made from the center of the umbilical to the lower edge of the umbilical wheel, and then, the self-made operation platform was implanted through the umbilicus. The external diameter of 10 mm and 5 mm instruments and camera lens were implanted at the finger end of the glove. After successfully entering the abdominal cavity, the pneumoperitoneum was established, the pressure was 12-14 (mmHg), the patient's body position was adjusted to 30°, the head was low, and the hip was high, so as to use the uterine lifting device. The pelvic cavity was evaluated by laparoscopy. Bipolar electrocoagulation was used to shorten the isthmus of the fallopian tube, the round ligament of the uterus, and the inherent ligament of the ovary, and then, the broad ligaments in the anterior and posterior parts and the peritoneal reflection of the bladder were opened, respectively. Bipolar electrocoagulation of bilateral uterine arteries and veins was performed. The cervical stump 1-10# absorption suture was selected to stop bleeding, and the uterus was removed at vertebral body and parallelly at the isthmus above the uterine vascular suture. After cervical reduction, the tract mucosa and pelvic peritoneum were sutured. Before the end of the operation, the pelvic wound was examined, and repeated washing was performed to stop bleeding. After incision suture, the operation ended.

Hardware platform: Ubuntu 16.04 operating system, deep learning framework is Pytorch-1.2.0. Python 3.6 is the development language, memory 128 GB, central processor is IntelXeon (R) Silver 4110CPU@2.10 GHz×32, and image processor is NVIDIA 1080Ti.

### 2.3. Observation Indicators

The intraoperative blood loss, postoperative pain score, postoperative fever, postoperative exhaust time, conversion operation, and operation time were recorded.

Pain degree: numerical rating scale (NRS) score was used (Table 1).

### 2.4. BCNN Structure

The BCNN structure is shown in Figure 1. In this algorithm, after optimizing the minimum loss, the two networks supervised each other, and it did not require a lot of time to adjust the parameters. Finally, the accurate recognition results were obtained. The parallel network of CNN Stream A and CNN Stream B extracted the cross-sectional features with high recognition in the input network image. The features extracted by CNN Stream A and CNN Stream B were fused, which helped to identify subtle features.

The image processing technology of deep learning used superimposing multiple convolutions to obtain image characteristics and then used multilayer perceptron to classify them. In clinical practice, the standard constrained deep network was used to realize the transverse section of ultrasound imaging. The doctor needed to spend a lot of experience in finding the horizontal transverse section during the examination, which was particularly important to have a standard access that can accurately identify the transverse section of the uterus. BCNN-S and BCNN-R were proposed to identify the transverse section of uterine ultrasound. First, image processing was performed, then the high transverse section was identified, and finally the features were fused. After obtaining the subtle features, the identification and classification were performed, and finally, the accurate identification of the horizontal direction of the transverse section of uterus was obtained.

The algorithm was optimized. The initial learning efficiency was set to 1, the weight attenuation was set to 1*e* − 5, the momentum attenuation was set to 0.9, and the learning rate of each epoch was multiplied by 0.1. The gradient was updated after algorithm optimization, which was more stable and smoother. The default parameters can make the model reach a stable level (Table 2).

### 2.5. Space Conversion Module

Through the attention mechanism, the space transformer networks (STN) can convert the spatial information in the original image to another space to retain key information. The spatial transformer (ST) was proposed. The spatial domain information in the image is transformed to extract key information. The trained STN can find out the areas that need to be concerned in the image information. ST has the function of scaling and rotation. The local information of the image can be extracted by transformation. ST module is input to the existing network structure. The model input equation is shown as follows.

(1) $$\begin{array}{c} Q\in R^{H\times W\times C}. \end{array}$$

*W* represents the width, *H* represents the height of the output tensor of the upper layer, and *C* represents the channel. Different convolution kernels and basic three channels of the image produce different channel information. The input image enters the double-stream route, and the transformed image is obtained through matrix change.

(2) $$\begin{array}{c} V^{\prime }\in R^{H\times W\times C}. \end{array}$$

*V*′ represents the transformed image features, and the positioning network learns a set of parameters *ϴ*. This parameter generates a sampling signal through the parameters of the grid generator, which is essentially the transformation of the matrix image.

The sampling matrix generated by STN can extract the key information in the original image. One is the sampling matrix for scaling and rotation transformation, and the other is the unit matrix, which is expressed as follows.

(3) $$\begin{array}{c} \left(\begin{array}{c} {X^{s}}_{i}\\ {Y^{s}}_{i} \end{array}\right)=T_{\theta }\left(Gi\right)={AZ}_{\theta }\left(\begin{array}{c} {X^{s}}_{i}\\ {Y^{s}}_{i}\\ 1 \end{array}\right)=\left(\begin{array}{c} \theta_{11}\theta_{12}\theta_{13}\\ \theta_{21}\theta_{22}\theta_{23} \end{array}\right)\left(\begin{array}{c} {X^{s}}_{i}\\ {Y^{s}}_{i}\\ 1 \end{array}\right). \end{array}$$

*ϴ* matrix is the corresponding sampling matrix. This module can identify the key information of the module on the upper layer. It is also a matrix that can be differentiated. It uses the kernel function to represent the complex change information.

(4) $$\begin{array}{c} {V^{\text{c}}}_{i}=\overset{H}{\underset{n}{\sum }}\overset{W}{\underset{m}{\sum }}{B^{c}}_{nm}T\left({x^{s}}_{i}-m;\psi x\right)*\left({y^{s}}_{i}-n;\psi y\right). \end{array}$$

*T* is the conversion kernel function, *B* represents the information before conversion, and *V* represents the information after conversion.

Classification network has strong feature representation ability and good recognition ability for conventional images. In target recognition, the difference between different targets is very small, but it is not ideal to classify directly in conventional images. In the debugging of fine-grained classification network, the loss measurement function is introduced. There will be three weight shared networks *q*, *m*, and *s* when three samples are input each time. The accumulated three network outputs obtain the loss, and in addition to the use of softmax loss function, the three characteristic outputs constitute the Triplet loss.

(5) $$\begin{array}{c} F=\lambda_{\text{s}}F_{s}\left(q\right)+\left(1-q\right)F_{t}\left(q,m,s\right). \end{array}$$

*F*_*s*_(*q*) represents the loss obtained by the softmax loss function, which represents the overall category information of the image so that the network can be optimized to the real category. *F*_*t*_(*q*, *m*, *s*) belongs to the Triplet error of three sub networks *f*_*q*_*s*, *f*_*m*_*s*, *f*_*s*_*s* with shared parameters. In order to increase the recognition ability of the same category and different samples of the network, the distance between classes is calculated. The two loss functions restrict each other, and the performance of the model is significantly improved.

When detecting the target, CNN can train through the object frame and component annotation in the fine-grained training image, including object head detection, fine-grained object level detection, and trunk detection. Ideal object detection results can be obtained by using position geometric constraints.

After the residual attention module can strengthen the attention and image features, the features are input into the next module at the same time. The *W*_*i*_, *c*(*x*) function represents different functions and has different attention domains. The equation is as follows.

(6) $$\begin{array}{c} W_{1}\left(x_{i,c}\right)=\frac{1}{1+\exp\left(-x_{i,c}\right)}, \end{array}$$

(7) $$\begin{array}{c} W_{2}\left(x_{i,c}\right)=\frac{x_{i,c}}{\left\|x_{i}\right\|}, \end{array}$$

(8) $$\begin{array}{c} W_{3}\left(x_{i,c}\right)=\frac{1}{1+\exp\left(-\left(x_{i,c}-\text{m}ean_{c}\right)/std_{c}\right)}. \end{array}$$

*W*_1_ indicates that the Sigmoid function directly activates the image feature tensor, *W*_2_ indicates that the image feature tensor is globally averaged and pooled to obtain channel domain attention, and *W*_3_ indicates the average number of Sigmoid functions activating the image feature tensor to obtain spatial domain attention.

### 2.6. Performance Evaluation Indicators

Reasonable evaluation of performance indicators can effectively evaluate the performance of the algorithm. The cross section of ultrasonic image is evaluated as a binary classification problem. The prediction category and real category of the model are divided into true negative (TN), false positive (FP), true positive (TP), and false negative (FN).

The accuracy calculation is shown in Equation (9). The higher the accuracy of classification, the better the performance of the algorithm. Precision refers to the proportion of TP in all samples predicted to be positive. Recall indicates the proportion of samples predicted to be positive in positive samples. When the recall rate and accuracy rate are high, the average will be higher. If one of them is low, it will lower the average, and its value will be close to the low number, as shown in Equation (12).

(9) $$\begin{array}{c} \text{Accuracy}=\frac{\text{TP}+\text{FN}}{\text{TP}+\text{FP}+\text{TN}+\text{FN}}, \end{array}$$

(10) $$\begin{array}{c} \text{Precision}=\frac{\text{TP}}{\text{TP}+\text{FP}}, \end{array}$$

(11) $$\begin{array}{c} \text{Recall}=\frac{\text{TP}}{\text{TP}+\text{FN}}, \end{array}$$

(12) $$\begin{array}{c} F1=\frac{2PR}{P+R}. \end{array}$$

It is required to make evaluation on the overall mean Intersection over Union (mIoU) and mean Dice of graph. mIoU predicts the intersection of the target area and the real target area. The higher the value of mIoU, the higher the correlation. mDICE is used to calculate the similarity between two samples. It is a geometric similarity measurement function. GT in Equation (14) denotes the true region, and Pre denotes the predicted region.

(13) $$\begin{array}{c} \text{IOU}=\frac{\text{GT}\cap \text{Pre}}{\text{GT}+\text{Pre}}, \end{array}$$

(14) $$\begin{array}{c} \text{DICE}=\frac{2\left|\text{GT}\cap \text{Pre}\right|}{\left|\text{GT}\right|+\left|\text{Pre}\right|}. \end{array}$$

The experimental environment hardware: platform memory (RAM) is 128 GB, the image processor (GPU) is NVIDIA 1080Ti ×2, the central processing unit (CPU) is Intel Xeon®Silver4110 CPU@2.10 GHz ×32, and the operating system is Ubuntu 16.04. The deep learning framework is Pytorch1.2.2, and Python 3.6 is selected as the development language.

### 2.7. Statistical Methods

The database of all data was established by Excel, and SPSS 19.0 statistical software was adopted. Measurement data were expressed as mean ± standard deviation ($\overset{¯}{x}\pm s$), enumeration data were analyzed by the *χ*^2^ test, and enumeration data were expressed as percentage (%). *P* < 0.05 was considered to indicate a significant difference.

## 3. Results

### 3.1. Training and Test Data Results

In this study, 3619 ultrasound images were obtained from the public dataset HC18 and the self-built dataset JFU19 after preprocessing, which were divided into training set and data set according to a certain proportion, and a certain number of training sets were drawn to evaluate the model, it was shown the model had a good recognition effect, and the three positions of horizontal, vertical, and right-angle lines were trained, respectively, and the results are shown in Figure 2. The test of the training set revealed that the model showed a good performance.

### 3.2. Parameter Information of BCNN

In this study, BCNN-R and BCNN-S feature images were extracted to analyze the performance of the algorithm. The resulting feature is shown in Figure 3. The feature image has distinct activation regions, which also indicates that there are many features that can be used for network identification and classification. Compared with BCNN-S B, BCNN-R A has more activated regions, which also obtains more identification ability. The ultrasound image in Figure 3(c) has more noise and reverberation than that in Figure 3(d). BCNN-R has a more complex structure and is inevitably subjected to a lot of noise.

### 3.3. Algorithm Performance Comparison

Comparing the algorithm performance of BCNN-R and BCNN-S with that in References [22–24], the highest accuracy of BCNN-S was 88.98%, followed by 85.62% of BCNN-R. BCNN-R had the highest recall rate of 88.51%, followed by BCNN-S of 87.54%; the highest accuracy of BCNN-R was 97.34%, followed by 91.67% of BCNN-S (Figure 4).

### 3.4. Experimental Results of Semantic Segmentation

In order to explore the change of the algorithm with epoch and the performance of the algorithm in ultrasonic image segmentation, the mIoU and mDICE evaluation indexes were analyzed. The results were as follows. Compared with mIoU and mDICE in Reference [24], mIoU and mDICE in BCNN had higher convergence performance, which can increase the robustness of the network to a certain extent and inhibit overfitting (Figure 5).

### 3.5. Ultrasound Results

The ultrasound parameters BNSD, CSD, PUA, bladder neck mobility, and BND under the maximum Valsalva state and at rest were compared between the two groups. It had a reduced BNSD under Valsalva state compared with that under at rest (Table 3).

### 3.6. Comparison of Surgical Conditions

The operation time, NRS score, intraoperative blood loss, and exhaust time of the two groups were compared. The operation time, intraoperative blood loss, and exhaust time of the two groups were similar, and the difference was not statistically significant (*P* > 0.05). In the NRS score, the pain of the observation group was mild, and the difference was significant (*P* < 0.05) (Table 4).

### 3.7. Comparison of Hospitalization Time and Satisfaction

The satisfaction score of the observation group was 5.32 ± 0.16, and that of the control group was 4.96 ± 0.21. The hospitalization time of the observation group was 6.72 ± 2.32 days, and that of the control group was 8.13 ± 2.18 days. The difference between the groups was statistically significant (*P* < 0.05) (Figure 6).

### 3.8. Postoperative Comparison

Abdominal infection, hematoma, incision bleeding, and incision infection did not occur in both groups after operation, and the patients recovered well. However, in the control group, one patient had active bleeding in the umbilical region after operation, and the dressing became dry after hemostasis with pressurized sand. The incidence of fever in the observation group was 1 case (2.5%), and that in the control group was 3 cases (7.5%). The fever rate in the control group was significantly higher than that in the observation group (*P* < 0.05) (Figure 7).

## 4. Discussion

Total hysterectomy is a relatively common gynecological surgery. After hysterectomy, the whole physiological state and overall structure of pelvic floor will change, which may produce PDF. Female pelvic floor is intricate, and it is important to find a noninvasive, reproducible, and simple diagnostic method for assessing pelvic floor function. With the rapid development of surgical abdominal surgery, LESS, with the natural approach, is widely used in clinical practice and is easier to understand and accept for some gynecological patients who meet the surgical criteria [25]. Compared with traditional hysterectomy, laparoendoscopic single-site total hysterectomy reduced hospital stay and postoperative blood loss, the two groups of patients had similar operation time, intraoperative blood loss, and exhaust time, and the difference had no statistical significance (*P* > 0.05); in the NRS score, the pain of the observation group was mild, and the difference had statistical significance (*P* < 0.05). Chung [26] compared single-site laparoscopic total hysterectomy with conventional laparoscopic total hysterectomy, there was no difference in pain scores between the two groups, and the operation time was significantly longer in single-site laparoscopic total hysterectomy group. In the observation group, intelligent algorithm was added in the ultrasound imaging, and there was no significant difference in the operation time. One patient had active bleeding at the umbilicus after surgery, and the dressing became dry after hemostasis with pressurized sand.

Ultrasonic technique of the BCNN model based on deep learning is accurate for evaluating pelvic floor function. Yu et al. [27] evaluated the effect of laparoscopic hysterectomy based on artificial intelligence imaging; ultrasound imaging based on ISCB algorithm can high-quality display the pelvic floor structure of patients undergoing total laparoscopic hysterectomy, improve the diagnostic rate of doctors, accelerate postoperative rehabilitation of patients, reduce postoperative pain, and improve patient satisfaction. In this experiment, BCNN-S had the highest accuracy of 88.98%; BCNN-R had the highest recall of 88.51%; and BCNN-R had the highest precision of 97.34%. The proposed algorithm shows high convergence performance in ultrasonic image segmentation. This experiment also shows that the intelligent algorithm of deep learning can effectively improve the efficacy of hysterectomy patients. Compared with mIoU and mDICE in Reference [24], mIoU and mDICE in BCNN had higher convergence performance, which can increase the robustness of the network to a certain extent and inhibit overfitting.

## 5. Conclusion

Eighty patients undergoing transumbilical single-site laparoscopic total hysterectomy in hospital were randomly divided into the treatment group and the control group to investigate the efficacy and safety of ultrasound based on deep learning for pelvic floor function in patients undergoing LESS. Ultrasound technology can be used to dynamically observe the anatomy of female pelvic floor organs; ultrasound technology of BCNN model based on deep learning has no significant toxic and side effects, with higher accuracy for evaluating the pelvic floor function. The incidence of pelvic floor dysfunction after hysterectomy is small, and attention should be paid to pelvic floor disorders and the image of sexual function during surgery, which is more conducive to the recovery of physical and mental health and normal life of patients. There are some shortcomings, due to the limitation of time, there is a lack of long-term follow-up, so long-term follow-up to patients is needed at a later stage to further verify the long-term efficacy. It is believed that it can provide some ideas and experimental support for the recovery of pelvic floor function in patients undergoing LESS.

## Figures and Tables

**Figure 1:** BCNN structure.

**Figure 2:** The comparison results between training set and test set. (a) The processing results of the public dataset HC8 for ultrasonic images. (b) The processing results of JFU19 for ultrasonic images.

**Figure 3:** BCNN-R and BCNN-S feature images. (a) The activation region shown in the BCNN-R feature image. (b) The activation region shown in the BCNN-S feature image. (c) The activation process of region classification by BCNN-R feature map. (d) The activation process of region classification by BCNN-S feature image.

**Figure 4:** Performance comparison of algorithms. (a) Comparison results of four algorithms in accuracy. (b) Comparison results of four algorithms in recall. (c) Comparison results of four algorithms in precision.

**Figure 5:** Performance comparison of algorithms. (a) The comparison between BCNN and UnetcsE algorithm in mDICE. (b) The comparison between BCNN and UnetcsE algorithm in mIoU.

**Figure 6:** Comparison of hospitalization time and satisfaction between the two groups. (a) Comparison result of hospitalization time between the two groups. (b) Satisfaction score of two groups. ^∗^Compared with the control group, *P* < 0.05.

**Figure 7:** Comparison of postoperative fever rate. ^∗^Compared with the control group, *P* < 0.05.

**Table 1:** NRS.

Score	Symptoms
0	Painless
1-3	Mild pain, sleep unaffected
4-6	Moderate pain, sleep affected
7-10	Severe pain, sleep affected seriously

**Table 2:** BCNN parameters.

Layer name	Kernel	Layer name	Kernel
	BCNN-R		BCNN-S
Conv 1	7 × 7, 64, stride 2	Conv 1	
Block 1	1 × 1, 64	Fire 1-3	1 × 1, 3 × 3, 64
	3 × 3, 64		1 × 1, 3 × 3, 64
	1 × 1,256		1 × 1, 3 × 3, 256
Block 2	1 × 1,128	Fire 4-7	1 × 1, 3 × 3, 256
	3 × 3,128		1 × 1, 3 × 3, 384
	1 × 1,512		1 × 1, 3 × 3, 512
Block 3	1 × 1,256		1 × 1, 3 × 3, 512
	3 × 3,256		
	1 × 1, 1024		
Block 4	1 × 1,512	Fire 8	2 × 2, maxpool, stride 2
	3 × 3,512		1 × 1, 3 × 3,512
	1 × 1, 2048		
Pool		Outer product	

**Table 3:** Result comparison between the two groups under at rest and Valsalva state.

Group	Number	BNSD	CSD	PUA	BND
Observation group	At rest	25.34 ± 3.12	31.87 ± 2.31	101.3 ± 8.41	7.12 ± 3.8
	Valsalva state	19.87 ± 4.5	32.7 ± 3.18	121.87 ± 12.6	8.7 ± 1.31
Control group	At rest	22.87 ± 2.8	31.87 ± 2.31	98.5 ± 7.86	6.1 ± 4.3
	Valsalva state	18.17 ± 2.31	30.87 ± 3.17	119.7 ± 9.38	8.67 ± 2.2

**Table 4:** Comparison of surgical conditions.

Group	Number	Operation time (min)	NRS cores	Exhaust time (h)	Intraoperative blood loss (ml)
Observation group	40	87.4 ± 9.76	1.87 ± 0.31^∗^	30.3 ± 2.41	112.1 ± 10.8
Control group	40	80.1 ± 8.3	2.29 ± 0.15	32.5 ± 1.86	153.1 ± 18.3
*P*		>0.05	<0.05	>0.05	>0.05

Note: ^∗^compared with the control group, *P* < 0.05.

## Data Availability

The data used to support the findings of this study are available from the corresponding author upon request.

## References

[1] Louis-Charles K., Biggie K., Wolfinbarger A., Wilcox B., Kienstra C. M. (2019). Pelvic floor dysfunction in the female athlete. *Current Sports Medicine Reports*.

[2] Ramdhan R. C., Loukas M., Tubbs R. S. (2017). Anatomical complications of hysterectomy: a review. *Clinical Anatomy*.

[3] Berghmans B. (2018). Physiotherapy for pelvic pain and female sexual dysfunction: an untapped resource. *International Urogynecology Journal*.

[4] Sendag F., Akdemir A., Zeybek B., Ozdemir A., Gunusen I., Oztekin M. K. (2014). Single-site robotic total hysterectomy: standardization of technique and surgical outcomes. *Journal of Minimally Invasive Gynecology*.

[5] Nam E. J., Kim S. W., Lee M. (2011). Robotic single-port transumbilical total hysterectomy: a pilot study. *Journal of Gynecologic Oncology*.

[6] Sinha R., Sundaram M., Mahajan C. (2010). Single-incision total laparoscopic hysterectomy. *Journal of Minimal Access Surgery*.

[7] Chen L., Zheng Y., Min L., Dong S. M. (2020). Clinical cohort study of total hysterectomy via transvaginal natural orifice transluminal endoscopic surgery and transumbilical laparoendoscopic single site surgery. *Zhonghua fu Chan ke za zhi*.

[8] Wallace S. L., Miller L. D., Mishra K. (2019). Pelvic floor physical therapy in the treatment of pelvic floor dysfunction in women. *Current Opinion in Obstetrics & Gynecology*.

[9] Lawson S., Sacks A. (2018). Pelvic floor physical therapy and women’s health promotion. *Journal of Midwifery & Women's Health*.

[10] Jung Y. W., Kim Y. T., Lee D. W. (2010). The feasibility of scarless single-port transumbilical total laparoscopic hysterectomy: initial clinical experience. *Surgical Endoscopy*.

[11] Prendergast S. A. (2017). Pelvic floor physical therapy for vulvodynia: a clinician’s guide. *Obstetrics and Gynecology Clinics of North America*.

[12] Chen S., Wang Y., Yang F., Wang K., Zheng Y. (2021). WITHDRAWN: Transumbilical laparoendoscopic single-site surgery (TU-LESS) extraperitoneal approach for lymphadenectomy: an innovative method. *Journal of Gynecologic Oncology*.

[13] Akdemir A., Yildirim N., Zeybek B., Karaman S., Sendag F. (2015). Single incision trans-umbilical total hysterectomy: robotic or laparoscopic?. *Gynecologic and Obstetric Investigation*.

[14] Cai H. H., Liu M. B., He Y. L. (2016). Treatment of early stage endometrial cancer by transumbilical laparoendoscopic single-site surgery versus traditional laparoscopic surgery: a comparison study. *Medicine (Baltimore)*.

[15] Huang L., He L., Zhang L. (2021). Application of the prone position in myomectomy by transvaginal natural orifice transluminal endoscopic surgery. *Videosurgery and Other Miniinvasive Techniques*.

[16] Saravelos S. H., Jayaprakasan K., Ojha K., Li T. C. (2016). Assessment of the uterus with three-dimensional ultrasound in women undergoing ART. *Human Reproduction Update*.

[17] Evans A. T., Szlachetka K., Thornburg L. L. (2019). Ultrasound assessment of the intrauterine device. *Obstetrics and Gynecology Clinics of North America*.

[18] Lv Z., Qiao L. (2020). Analysis of healthcare big data. *Future Generation Computer Systems*.

[19] Xie S., Yu Z., Lv Z. (2021). Multi-disease prediction based on deep learning: a survey. *Computer Modeling in Engineering & Sciences*.

[20] Yu Z., Amin S. U., Alhussein M., Lv Z. (2021). Research on disease prediction based on improved DeepFM and IoMT. *IEEE Access*.

[21] Choi Y. S., Park J. N., Oh Y. S., Sin K. S., Choi J., Eun D. S. (2013). Single-port vs. conventional multi-port access laparoscopy-assisted vaginal hysterectomy: comparison of surgical outcomes and complications. *European Journal of Obstetrics & Gynecology and Reproductive Biology*.

[22] Tobias-Machado M., Chicoli F. A., Costa Jr R. M. (2012). LESS sacrocolpopexy: step by step of a simplified knotless technique. *International braz j urol*.

[23] Huang G., Liu Z., Pleiss G., Van Der Maaten L., Weinberger K. (2019). Convolutional networks with dense connectivity. *IEEE Transactions on Pattern Analysis and Machine Intelligence*.

[24] Toussaint N., Khanal B., Sinclair M. (2018). Weakly supervised localization foe fetal ultrasound images. *Deep Learning in medical image analysis and multimodal learning fo clinical decision support*.

[25] Oh S. J., Lee S. Y., Kim W. Y. (2020). Comparison between transumbilical and transvaginal morcellation of a large uterus during single-port-access total laparoscopic hysterectomy. *Obstetrics & Gynecology Science*.

[26] Chung J. H., Baek J. M., Chung K. (2015). A comparison of postoperative pain after transumbilical single-port access and conventional three-port total laparoscopic hysterectomy: a randomized controlled trial. *Acta Obstetricia et Gynecologica Scandinavica*.

[27] Yu H., Zhao Z., Duan X., Zhou J., Su D. (2022). Ultrasound image under artificial intelligence algorithm to evaluate the intervention effect of accelerated rehabilitation surgery nursing on laparoscopic hysterectomy. *Computational Intelligence and Neuroscience*.

